# Effect of Different Anesthesia Methods on Emergence Agitation and Related Complications in Postoperative Patients with Osteosarcoma

**DOI:** 10.1155/2021/7120035

**Published:** 2021-12-14

**Authors:** Minghuan Zhang, Bo Wang, Wen Mao

**Affiliations:** ^1^Department of Orthopedics,Guanggu Hospital Area, Wuhan Third Hospital, Wuhan 430071, Hubei Province, China; ^2^Department of Anesthesiology,Guanggu Hospital Area, Wuhan Third Hospital, Wuhan 430071, Hubei Province, China

## Abstract

**Purpose:**

To explore the effect of different anesthesia methods on emergence agitation (EA) and related complications in postoperative patients with osteosarcoma.

**Methods:**

According to the order of admission, 115 patients requiring osteosarcoma surgery treated in our hospital from January 2018 to December 2020 were selected as the research object and randomly divided into the control group (*n* = 57, accepted the general anesthesia with tracheal intubation) and the experimental group (*n* = 58, accepted the combined spinal-epidural anesthesia) to compare their anesthesia effect, incidence rates of agitation and complications, and other indexes.

**Results:**

In terms of the hemodynamic indexes (MAP, HR, and CVP values), both groups had lower ones at *T*_1_ than at *T*_0_, but the decline of the experimental group was generally lesser than that of the control group; at *T*_2_, no statistical difference was shown within the experimental group's indexes when comparing with those at *T*_1_, but the control group obtained a significant increase; at *T*_3_ and *T*_4_, both groups had their hemodynamic indexes increased, but such increase within the experimental group showed no statistical difference when comparing with those at *T*_0_, while the control group achieved obviously higher values at *T*_4_ than at *T*_0_ (before the anesthesia); and the between-group difference in the hemodynamic indexes at *T*_1_ and *T*_4_ was significant. Compared with the control group, the experimental group achieved better VAS scores and anesthesia indexes and lower incidence rates of EA and complications such as the hypoxemia, cardiovascular response, delayed recovery, and headache. In addition, the differences in the incidence rates of hypotension and cognitive dysfunction between the two groups were not statistically significant.

**Conclusion:**

When comparing with tracheal intubation general anesthesia, the combined spinal-epidural anesthesia has a better effect in osteosarcoma surgery, with less hemodynamics influence on patients, reduced postoperative pain and stress reaction, and lowered incidence rates of postoperative EA and complications, which is worthy of wide application in clinical treatment.

## 1. Introduction

Osteosarcoma is a malignant bone tumor that involves the cortical bone, marrow cavity, and periosteum and usually occurs in proximal tibia, proximal humerus, and metaphysis of the distal femur by the way of directly producing osteoid tissue with tumor cells. It is often presented as grayish-red or brownish-red spindle-shaped tumor with fish-like lesion section [1–4]. The main symptom of osteosarcoma is persistent local pain, which may be aggravated with the condition getting more serious, especially at night, and accompanied with local masses in patients with severe condition, leading to limited movement of peripheral joints. In addition, increased temperature and venous engorgement are often shown on the local skin. According to relevant statistics, about 60% osteosarcoma patients are under the age of 25, and the incidence rate is much higher in men than in women with the male-female ratio of 3 : 2 [5–8]. The causes for the abnormal proliferation of the malignant tumor cells are unknown. Currently, the treatment plan for osteosarcoma mainly covers preoperative chemotherapy, surgical resection, and postoperative chemotherapy, of which surgical resection is the critical part with the main aim being complete resection of lesion and preservation of limb function as far as possible [9–12]. Clinically, general anesthesia patients in the awakening period may be irritated by operations such as tracheal intubation and suctioning and thus are prone to increased heart rate and blood pressure, which may further cause agitation and seriously affect the postoperative rehabilitation effect. Therefore, the way of controlling emergence agitation (EA) after anesthesia has always been a research hotspot of clinical surgery. Combined spinal-epidural anesthesia is an emerging anesthesia modality in recent years, which has advantages such as the fast onset and good blocking effect. In addition, it ensures prolonged surgical anesthesia, which meets the demand of osteosarcoma surgery, but there are few related studies currently. To solve the problem fundamentally, the effect of different anesthesia methods on EA and related complications in postoperative patients with osteosarcoma was explored, and the summary results are as follows.

## 2. Materials and Methods

### 2.1. General Information

115 patients with the need of osteosarcoma surgery treated in our hospital from January 2018 to December 2020 were selected as the research object and randomly divided into the control group (*n* = 57) and the experimental group (*n* = 58) according to the order of admission. The comparison result of the baseline information of patients between the two groups showed no statistical significance (*P* > 0.05) and no influence on the study of between-group difference (Table 1).

### 2.2. Inclusion Criteria

The inclusion criteria were as follows: patients met the relevant indicators of osteosarcoma surgery; the American Society of Anesthesiologists (ASA) grades were I–III; patients had no history of relevant drug allergies; patients had no mental or other cognitive impairment; and the study was approved by the hospital ethics committee, and patients' family members signed the informed consent.

### 2.3. Exclusion Criteria

The exclusion criteria were as follows: suffering from osteosarcoma combined with other serious diseases of the brain, heart, kidney, and liver; taking sedative medications chronically; with excessive surgical time (>3 h); refusal to cooperate with the study; and in the gestation period or lactation period.

## 3. Methods

Patients in both groups fasted for 8 hours before surgery. After entering the operating room, patients had their venous passage opened and inhaled oxygen, and their ECG, pulse, and oxygen saturation were monitored, as well as their mean arterial pressured (with radial artery catheterization) and central venous pressure (with venipuncture catheter in the right neck) before implementation of anesthesia.

Control group (under general anesthesia): after intravenous infusion of 0.3 *µ*g kg^−1^ h^−1^ sufentanil and 4 mg kg^−1^ h^−1^ propofol, patients fell asleep and underwent induction intubation by injecting 0.15 mg/kg of cisatracurium intravenously, which was added during the surgery to maintain appropriate muscle tone.

Experimental group (under combined spinal-epidural anesthesia): before anesthesia, 0.3 *µ*g kg^−1^ h^−1^ sufentanil and 4 mg kg^−1^ h^−1^ propofol were injected intravenously for sedation and analgesia [13–16]. Patients were kept in lateral position with the affected limb upward, the spinal L_2-3_ or L_3-4_ space was selected as the puncture point, routine disinfection and drape were performed, the infiltrated point was under local anesthetic, and after breaking through the ligamentum flavum, the spinal needle was inserted; when the cerebrospinal fluid flowed out, 2-3 ml 0.5% ropivacaine was injected, the spinal needle was withdrawn, the epidural catheter was inserted, and the fixation was performed after there was no cerebrospinal fluid and blood when pumping back. During the surgery, 0.5% ropivacaine could be given repeatedly and in small amount through the epidural catheter according to patients' condition. Patients in both groups were given 4 mg kg^−1^ h^−1^ propofol by intravenous injection during the surgery to maintain appropriate sedation depth.

### 3.1. Observation Indexes

Hemodynamic indexes: the mean arterial pressure (MAP), heart rate (HR), and central venous pressure (CVP) of patients in both groups were monitored in the following time points: before anesthesia (*T*_0_), after completion of anesthesia (*T*_1_), the start of surgery (*T*_2_), the end of surgery (*T*_3_), and the end of anesthesia (*T*_4_).

VAS score: patients' physical pain was evaluated by the visual analog scale (VAS), with 0 point indicating no pain, 3 points or less indicating slight pain, 4–6 points indicating tolerable pain but the patient's sleep is affected, and 7–10 points indicating intolerably strong pain that seriously affects the patient's sleep and appetite.

Anesthesia indexes included the anesthesia onset time, motor block recovery time, sensory block recovery time, and postoperative awake time.

Grade of EA: grade 0 (no agitation) meant the patient cooperated quietly; grade I (slight agitation) meant the patient groaned intermittently; grade II (mild agitation) meant the patient groaned constantly; and grade III (severe agitation) meant the patient screamed and struggled unremittingly.

Complications included hypoxemia, hypotension, cardiovascular response, delayed recovery, cognitive dysfunction, and headache.

### 3.2. Statistical Processing

In this study, the data processing software was SPSS20.0, the picture drawing software for data was GraphPad Prism 7 (GraphPad Software, San Diego, USA), items included were enumeration data and measurement data, methods used were the *X*^2^ test, *t*-test, and normality test, and differences were considered statistically significant at *P* < 0.05.

## 4. Results

### 4.1. Comparison of Hemodynamic Indexes between the Two Groups

In terms of the hemodynamic indexes (MAP, HR, and CVP values), both groups had lower ones at *T*_1_ than at *T*_0_, but the decline of the experimental group was generally lesser than that of the control group; at *T*_2_, no statistical difference was shown within the experimental group's indexes when comparing with those at *T*_1_, but the control group obtained a significant increase; at *T*_3_ and *T*_4_, both groups had their hemodynamic indexes increased, but such increase within the experimental group showed no statistical difference when comparing with those at *T*_0_, while the control group achieved obviously higher values at *T*_4_ than at *T*_0_ (before the anesthesia); and the between-group difference in the hemodynamic indexes at *T*_1_ and *T*_4_ was significant (Figures 1–3).

### 4.2. Comparison of VAS Scores between the Two Groups

The VAS scores on pain of patients in the experimental group were significantly lower than those of the control group (*P* < 0.05), with statistically significant difference (Figure 4).

### 4.3. Comparison of Anesthesia Indexes between the Two Groups

The anesthesia indexes of the experimental group were significantly better than those of the control group (*P* < 0.05), with statistical differences (Table 2).

### 4.4. Comparison of Incidence Rates of EA between the Two Groups

The incidence rate of EA of the experimental group was significantly lower than that of the control group (*P* < 0.05), with a statistically significant difference (Table 3).

### 4.5. Comparison of Incidence Rates of Complications between the Two Groups

The incidence rates of hypoxemia, cardiovascular response, delayed recovery, headache, and other complications of the experimental group were significantly lower than those of the control group (*P* < 0.05), while there was no statistical difference in the incidence rates of hypotension and cognitive dysfunction between the two groups (*P* > 0.05) (Table 4).

## 5. Discussion

EA, a long-term focus in the field of clinical treatment, is a common adverse effect after anesthesia that causes sympathetic excitation and leads to increased blood pressure and lack of oxygen to the brain. In addition, as it is also a poor manifestation of mental disorders, patients with it mainly show illogical thought, psychic inadequacy, often some involuntary behaviors, and even mania in severe cases, which will not only make the postoperative work of medical and nursing staff more difficult but also change the hemodynamic indexes of patients and even form patients' tendency to violence such as spontaneous extubation. EA is detrimental to patients' physical recovery for it greatly reduces the compliance with treatment and easily leads to various postoperative complications [17–20]. There are many reasons why patients develop EA from anesthesia, but postoperative pain is the main one. Patients after osteosarcoma surgery often suffer from severe pain that will increase the content of aldosterone, catecholamine, and other substances in the body, leading to a rapid heartbeat and possible cardiovascular diseases [13, 21, 22]. Therefore, the effect of different anesthesia methods on postoperative EA and related complications are mainly investigated by retrospectively analyzing the clinical medical records of 115 patients requiring osteosarcoma surgery in our hospital.

The study first focused on the influence of general anesthesia with tracheal intubation and combined spinal-epidural anesthesia on the perioperative hemodynamic indexes (MAP, HR, and CVP values) and concluded that both groups had lower ones at *T*_1_ than at *T*_0_, but the decline of the experimental group was generally lesser than that of the control group, which was consistent with the report by Kumar [23]; at *T*_2_, no statistical difference was shown within the experimental group's indexes when comparing with those at *T*_1_, but the control group obtained a significant increase; at *T*_3_ and *T*_4_, both groups had their hemodynamic indexes increased, but such increase within the experimental group showed no statistical difference when comparing with those at *T*_0_, while the control group achieved obviously higher values at *T*_4_ than at *T*_0_ (before the anesthesia); and the between-group difference in the hemodynamic indexes at *T*_1_ and *T*_4_ was significant. The results presented the influence of the two anesthesia methods on patients' perioperative stress reaction, i.e., appropriate local anesthesia performed to the patients in the experimental group after the completion of general anesthesia could easily control the anesthetic plane to a suitable level, and although they achieved lower hemodynamic indexes, the decrease was slight, and they restored to normal after the end of anesthesia; however, due to the preoperative fasting required in the control group, lack of circulation and use of induced drug conferred a state of cardiovascular depression in patients. During surgery, as patients in the experimental group had their anesthesia plane fixed and their motor and sensory nerves innervating the surgical area blocked completely, a satisfactory and painless surgical environment with muscle relaxation was presented, and a small amount of drug could be given repeatedly through the epidural catheter with the analgesic and sedative effects lasted until patients regain consciousness, thereby relieving circulatory depression; in the control group, due to the fact that surgical skin incision produced a corresponding stress response, various vital signs were significantly elevated, which, combined with operations such as suturing skin at the end of the surgery and the extraction of the endotracheal tube after anesthesia, would cause hemodynamic indexes to rise rapidly and fluctuate in a large range. In addition, the VAS scores and anesthesia indexes of the experimental group were significantly better than those of the control group, the incidence rates of EA and complications such as hypoxemia, cardiovascular response, delayed recovery, and headache in the experimental group were significantly lower than those of the control group, and there was no significant between-group difference in the incidence rates of hypotension and cognitive dysfunction, indicating that the combined spinal-epidural anesthesia had a better effect and lower incidence rates of postoperative complications, which was of significant value and meaning to improve the prognosis effect. This study is consistent with the conclusion made by Smith et al. [16]. Compared with general anesthesia, combined spinal-epidural anesthesia can effectively reduce the incidence rates of EA after anesthesia as well as complications while maintaining stable hemodynamic indexes in patients undergoing osteosarcoma surgery and has higher safety.

In conclusion, when comparing with tracheal intubation general anesthesia, combined spinal-epidural anesthesia has exact efficacy, unlimited anesthesia time, small dose of local anesthetic, low incidence rate of poisoning by local anesthetic, and postoperative epidural analgesic effect, truly realizing the “noncontact” lumbar anesthesia technology. It has a better effect in osteosarcoma surgery, with less hemodynamics influence on patients, reduced postoperative pain and stress reaction, lowered incidence rates of postoperative EA and complications, and better anesthesia indexes, which is worthy of wide application in clinical treatment. However, as it was a single-center study with small sample size, the anesthesia management effect shall be comprehensively observed and applied, and a multicenter study with large sample size shall be conducted for further confirmation.

## Figures and Tables

**Figure 1:** Comparison of MAP between the two groups (‾*x* ± *s*). The horizontal axis indicates the time points and the vertical axis indicates the MAP level in mmHg; The MAP of the control group at *T*_0_, *T*_1_, *T*_2_, *T*_3_, and *T*_4_ was (78.15 ± 8.46), (72.13 ± 5.16), (75.21 ± 6.17), (76.52 ± 3.65), and (82.29 ± 8.15), respectively. The MAP of the experimental group at *T*_0_, *T*_1_, *T*_2_, *T*_3_, and *T*_4_ was (80.04 ± 6.25), (78.26 ± 5.33), (76.23 ± 6.14), (76.84 ± 6.17), and (77.14 ± 6.61), respectively. ^*∗*^ from left to right indicates that the differences in MAP at *T*_1_ and *T*_4_ between the two groups were significant (*t* = 6.2647, 3.7248; *P* < 0.001, *P*=0.0003). & indicates that the difference in MAP at *T*_0_ and *T*_1_ within the control group was significant (*t* = 4.6158, *P* < 0.001). && indicates that the difference in MAP at *T*_1_ and *T*_2_ within the control group was significant (*t* = 2.9059, *P*=0.0044). &&& indicates that the difference in MAP at *T*_0_ and *T*_4_ within the control group was significant (*t* = 2.6728, *P*=0.0086).

**Figure 2:** Comparison of HR between the two groups (‾*x* ± *s*). The horizontal axis indicates the time points and the vertical axis indicates the HR in times/min. The HR of the control group at *T*_0_, *T*_1_, *T*_2_, *T*_3_, and *T*_4_ was (76.59 ± 8.63), (67.89 ± 6.08), (70.05 ± 5.34), (74.21 ± 4.32), and (82.25 ± 6.48), respectively. The HR of the experimental group at *T*_0_, *T*_1_, *T*_2_, *T*_3_, and *T*_4_ was (76.45 ± 8.95), (72.31 ± 6.15), (71.43 ± 5.27), (73.61 ± 5.45), and (75.17 ± 6.11), respectively. ^*∗*^ from left to right indicates that the differences in HR at *T*_1_ and *T*_4_ between the two groups were significant (*t* = 3.8752, 6.0293; *P*=0.0002, *P* < 0.001). & indicates that the difference in HR at *T*_0_ and *T*_1_ within the control group was significant (*t* = 6.2583, *P* < 0.001). && indicates that the difference in HR at *T*_1_ and *T*_2_ within the control group was significant (*t* = 2.0228, *P*=0.0455). &&& indicates that the difference in HR at *T*_0_ and *T*_4_ within the control group was significant (*t* = 3.9817, *P* < 0.001).

**Figure 3:** Comparison of CVP between the two groups (‾*x* ± *s*). The horizontal axis indicates the time points and the vertical axis indicated the CVP level in cmH_2_O. The CVP of the control group at *T*_0_, *T*_1_, *T*_2_, *T*_3_, and *T*_4_ was (8.46 ± 0.37), (7.97 ± 0.46), (8.23 ± 0.65), (8.25 ± 0.92), and (8.71 ± 0.38), respectively. The CVP of the experimental group at *T*_0_, *T*_1_, *T*_2_, *T*_3_, and *T*_4_ was (8.48 ± 0.38), (8.26 ± 0.35), (8.25 ± 0.37), (8.32 ± 0.34), and (8.44 ± 0.33), respectively. ^*∗*^ from left to right indicates that the differences in CVP at *T*_1_ and *T*_4_ between the two groups were significant (*t* = 3.8088, 4.0704, *P*=0.0002, *P* < 0.001). & indicates that the difference in CVP at *T*_0_ and *T*_1_ within the control group was significant (*t* = 6.2998, *P* < 0.001). && indicates that the difference in CVP at *T*_1_ and *T*_2_ within the control group was significant (*t* = 2.4721, *P*=0.0149). &&& indicates that the difference in CVP at *T*_0_ and *T*_4_ within the control group was significant (*t* = 3.5737, *P*=0.0005).

**Figure 4:** Comparison of VAS scores on pain between the two groups (‾*x* ± *s*). The horizontal axis indicates the VAS score, and the vertical axis indicates the values. The VAS score on pain of the control group was (5.52 ± 1.23). The VAS score on pain of the experimental group was (1.92 ± 0.04). ^*∗*^The difference in the VAS scores on pain between the two groups was significant (*t* = 22.2798, *P* < 0.0001).

**Table 1:** Baseline information.

Category	Control group (*n* = 57)	Experimental group (*n* = 58)	t/*X*^2^	*P*
Age (years)	23.4 ± 4.8	22.9 ± 4.2	0.5200	0.6044
Weight (kg)	64.8 ± 7.9	65.4 ± 8.1	0.3518	0.7259
Surgery time (min)	102.4 ± 11.6	103.1 ± 11.3	0.2867	0.7750
Anesthesia time (min)	138.5 ± 15.4	139.7 ± 16.8	0.3493	0.7277
Gender				

Male	34 (59.65%)	36 (62.07%)	0.0707	0.790
Female	23 (40.35%)	22 (37.93%)		

ASA grade				
I	11 (19.30%)	13 (22.41%)	0.1690	0.681
II	22 (38.60%)	21 (36.21%)	0.0701	0.791
III	24 (42.11%)	24 (41.38%)	0.0062	0.937

**Table 2:** Comparison of anesthesia indexes between the two groups (‾*x* ± *s*, min).

Index	Control group (*n* = 57)	Experimental group (*n* = 58)	*t*	*P*
Anesthesia onset time	16.8 ± 2.5	5.7 ± 1.6	28.4092	<0.001
Motor block recovery time	234.5 ± 17.3	130.2 ± 14.8	34.7613	<0.001
Sensory block recovery time	213.1 ± 12.7	154.3 ± 11.7	25.8293	<0.001
Postoperative awake time	7.8 ± 1.2	3.1 ± 1.1	21.9008	<0.001

**Table 3:** Comparison of incidence rates of EA between the two groups (*n*(%)).

Grade	Control group (*n* = 57)	Experimental group (*n* = 58)	*t*	*P*
0	36 (63.16)	50 (86.21)		
I	13 (22.81)	5 (8.62)		
II	5 (8.77)	2 (3.45)		
III	3 (5.26)	1 (1.72)		
Total incidence rate	21 (36.84)	8 (13.79)	8.0986	0.004

**Table 4:** Comparison of incidence rates of complications between the two groups ((*n*(%)).

Complication	Control group (*n* = 57)	Experimental group (*n* = 58)	*t*	*P*
Hypoxemia	16 (28.07)	2 (3.45)	13.2008	<0.001
Hypotension	4 (7.02)	5 (8.62)	0.4009	0.527
Cardiovascular response	13 (22.81)	1 (1.72)	11.9512	0.001
Delayed recovery	17 (29.82)	0 (0)	20.2990	<0.001
Cognitive dysfunction	21 (36.84)	19 (32.76)	0.2113	0.646
Headache	8 (14.04)	2 (3.45)	4.0583	0.044

## Data Availability

The data used to support the findings of this study are available from the corresponding author upon request.
